RETRACTED

# Molecular Mechanism of Secondary Endocrine Resistance in Luminal Breast Cancer

**DOI:** 10.1155/2021/6618519

**Published:** 2021-03-16

**Authors:** Minhua Wu, Jinhua Ding, Limu Wen, Yuxin Zhou, Weizhu Wu

**Affiliations:** ^1^Li Huili Hospital, Ningbo Medical Center, Ningbo 315040, China; ^2^Medical School of Ningbo University, Ningbo 315040, China

## Abstract

**Objective:**

The molecular mechanism of secondary resistance in Luminal breast cancer was studied to provide new ideas for the treatment of breast cancer.

**Methods:**

The sensitivity of the downregulation of myeloid leukemia factor 1-interacting proteins (MLF1IP) to Tamoxifen (TAM) was tested by the Cell Counting Kit-8 (CCK-8). The apoptosis of MLF1IP-mediated resistance was analyzed by flow cytometry (FCM) with/without TAM. Western blot was used in detecting various kinds of apoptosis and the expression of the protein related to the phosphatidylinositol 3-kinase (PI3K)/AKT signaling pathway to study the molecular mechanism of secondary endocrine resistance in Luminal breast cancer.

**Results:**

The downregulation of MLF1IP could significantly increase the drug sensitivity of Michigan Cancer Foundation-7 (MCF-7) cells and also inhibit the proliferation of MCF-7 cells under the stimulation of drugs. Western blot results showed that the expression of Bcl-2-associated X (BAX), Caspase3, Caspase7, and Caspase9 proteins increased when MLF1IP was downregulated. The results of the PI3K/AKT signaling pathway revealed that the phosphatase and tensin homolog deleted on chromosome ten (PTEN) protein expression of MCF7-shRNA was higher than that of MCF7-NC cells, while the expression of p-AKT was lower than that of MCF7-NC cells.

**Conclusions:**

(1) MLF1IP-related apoptosis resistance plays an essential role in MLF1IP-mediated secondary resistance of breast cancer cells. (2) MLF1IP promotes AKT phosphorylation by inhibiting the PTEN expression, thus activating the PI3K/AKT signaling pathway and causing the secondary resistance of Luminal breast cancer. (3) MLF1IP can be used as a factor to predict the endocrine resistance of Luminal breast cancer.

## 1. Introduction

According to statistics, nearly 1.7 million new breast cancer cases are diagnosed every year across the world, accounting for a quarter of malignant tumors in women. More than half a million women worldwide die of breast cancer every year [1, 2]. The incidence rate of breast cancer is increasing. Breast cancer has become one of the most common malignant tumors in modern women and severely affects women's health and life [3]. With the development of molecular biology, the research goes deep into breast cancer. Some research reports suggest that some molecules play a crucial part in the occurrence and development, invasion and metastasis, diagnosis, and treatment of breast cancer, such as estrogen receptor (ER), progesterone receptor (PR), and human epidermal growth factor 2 (HER-2) [4, 5]. ER-positive breast cancer accounts for the largest proportion of all breast cancer, reaching 70%. According to the molecular classification, ER-positive breast cancer can be divided into Luminal A and Luminal B [6]. Different treatments are used in patients with different breast cancers. Endocrine therapy (ET), as the primary treatment to breast cancers, can effectively reduce the recurrence rate and mortality of breast cancer. Tamoxifen (TAM) is the main drug in endocrine therapy for Luminal breast cancer, but some patients have resistance to it. The resistance, either primary or secondary, will influence the follow-up treatment, which, as a result, may cause the recurrence [7]. Therefore, the primary or secondary endocrine resistance, a significant problem in the clinical treatment of breast cancer, needs to be solved quickly to improve the life quality of those patients.

RETRACTED

The previous study shows that myeloid leukemia factor 1-interacting proteins (MLF1IP) is involved in the development of several kinds of tumors. Huang and Luo (2016) found that MLF1IP overexpression mattered much in the progress of Luminal breast cancer [8]. Yang et al. (2017) found that MLF1IP may contribute to the carcinogenic potential of breast cancer [9]. The study has proved that MLF1IP plays a vital part in endocrine resistance of breast cancer treatment, but its specific molecular mechanism is unknown.

To sum up, Luminal breast cancer is the most common, and endocrine therapy is the primary treatment, to which some patients will have secondary endocrine resistance. MLF1IP counts much in the endocrine resistance, but the specific molecular mechanism remains unclear. Therefore, the molecular mechanism of secondary endocrine resistance in Luminal breast cancer was studied using MLF1IP.

## 2. Materials and Methods

### 2.1. Experimental Materials

Michigan Cancer Foundation-7 (MCF-7) cell lines with high expression of MLF1IP were selected to study the molecular mechanism of secondary endocrine resistance in Luminal breast cancer. The selected MCF-7 was from American Type Culture Collection (ATCC). Roswell Park Memorial Institute- (RPMI-) 1640 medium containing 10% fetal bovine serum was used to culture for 48-72 h in 5% CO_2_ incubator at 37°C, and then 0.05% trypsin enzyme-digesting was used to transfer.

### 2.2. Real-Time Polymerase Chain Reaction (PCR)

The cells were lysed with TRIzol reagent (Invitrogen Biotechnology Co., Ltd., USA) and then separated by chloroform (Invitrogen Biotechnology Co., Ltd., USA). The upper colorless aqueous phase liquid was put into EP tube (Shanghai Yiheng Scientific Instrument Co., Ltd., China), and the equal volume of isopropanol (Invitrogen Biotechnology Co., Ltd., USA) was added for precipitation. Later, the cells were washed with ethanol. After the residual liquid was sopped up, the cells were dried and precipitated at room temperature. When the precipitation was almost transparent, ribonucleic acid (RNA) enzyme (Invitrogen Biotechnology Co., Ltd., USA) was added and dissolved. Then the concentration was determined by the multimode reader (Tecan Company, Switzerland). According to the designed reverse transcription system, reverse transcripts were detected immediately by real-time PCR.

RETRACTED

### 2.3. Cell Counting Kit-8 (CCK-8)

The culture solution and cells in the medium were transferred to a 15 mL centrifuge tube (Shanghai Yiheng Scientific Instrument Co., Ltd., China), centrifuged at 800 rpm for 5 min. Then, the supernatant was removed, and fresh medium was added. The counting started after the specimen was blown evenly. Then, the specimen was placed in an orifice plate (Corning Company, USA) in a 0.5% CO_2_ incubator (Thermo Scientific Company, USA) overnight at 37°C. The next day, TAM (4-hydroxyta, TAM reagent, purity ≥ 99.0%, Sigma Company, USA) was added into the cells according to the dilution ratio. At the same time, three repeated experiments were performed at each gradient. After 48 h, 10 *μ*L CCK (Dojindo Laboratories, Japan) was added into the corresponding pores. After the incubation at 37°C for 2 h, the absorbance (OD_450_) was determined at 450 nm. The data were analyzed. Then the mean value and the standard deviation of each concentration were taken by the multimode reader. In addition, the chart was made to calculate the *P* value.

### 2.4. Annexin V-APC/7-AAD

The culture solution containing cells was aspirated and placed in a 15 mL centrifuge tube. Centrifugation was performed at 800 rpm for 5 min. The supernatant was removed, and fresh culture medium was added. The counting started after the specimen was shaken evenly. The cells were cultured overnight in a 6-well plate at 37°C in 5% CO_2_ incubator. The next day, 32 *μ*M TAM was used. The supernatant of cell culture was collected and placed in a centrifuge tube of 3 independent experiments run in duplicate, and then centrifuged at 1500 rpm for 5 min. Later, the supernatant was removed, and the cells were washed with phosphate buffer solution (PBS) (Fuzhou Maixin Biotechnology Development Co., Ltd., China) and again centrifuged at 1500 rpm for 5 min to collect the cells. Then the specimen was washed and precipitated with binding buffer (TAKARA Biotechnology Co., Ltd., Japan), centrifuged at 1500 rpm for 5 min, and then the cells were collected. The cells were resuspended and precipitated with a 1 mL standing buffer. Then 100 *μ*L cell suspension was added into 5 *μ*L Annexin V-APC/7-AAD staining, and the cells were kept away from light for 10-15 min at room temperature. Finally, the samples were transferred to the flow tube (Corning company, USA) for detection.

RETRACTED

### 2.5. Western Blot Trial

The cells were collected into a 1.5 mL polypropylene tube (EP tube), and 4°C precooled protein lysate (Sigma Company, USA) was added to lyse for 30 min. The specimen was centrifuged at 4°C at 13,200 rpm for 15 min, and the supernatant was taken for standby. 98 *μ*L PBS was put into a new 1.5 mL EP tube, and a 2 *μ*L sample pyrolysis solution was added to mix the specimen well. 20 *μ*L sample was taken out and put into the 96-well plate, adding a 200 *μ*L BCA (Sigma Company, USA) working solution. The specimen was incubated at 37°C for 30 min. The multimode reader determined the absorbance of the sample diluted 50 times. The corresponding protein concentration was calculated on the standard curve. Later, the actual concentration of the sample was obtained by multiplying the sample dilution degree. The glass plate was fixed on the electrophoresis tank, 10% separating glue was prepared, and TEMED (Bio-Rad Company) was added. The glue was poured quickly and covered with water isobutanol. After separating glue aggregated 30 min, the covering liquid was poured out and washed with ddH_2_0 (Tecan Company, Switzerland) at the top of the gel for several times to remove unpolymerized acrylamide, and then the residual liquid was absorbed with absorbent paper. The prepared glue was quickly poured in, and the defoaming treatment was carried out at the same time. When the gel polymerized about 30 min, it was added into the electrophoresis tank. Afterward, the electrophoresis buffer was added. The protein sample and the treatment solution were mixed in EP tube, heated at 95°C for 10 min, and centrifuged after cooling in an ice bath. Protein was added to each well. The same amount of sample buffer was added into the sample hole to prevent edge effect. When the electrode plug was connected with a suitable electrode, the voltage was adjusted to 80 V. The front edge of the sample was moved about 40 min. When the voltage was changed to 120 V, the front edge of the sample was moved to the bottom. After the power was switched off, the gel glass plate was removed from the electrophoresis tank, and the spacers between the two fast glass plates were moved carefully. The spacers were inserted into the glass plate and gently pried open the glass plate to remove the stacking gel pasted on the groove and the hole adding no sample.

RETRACTED

### 2.6. Statistical Analysis

SPSS 22.0 was used for statistical analysis. The data of normal distribution were analyzed by *t*-test or analysis of variance, the comparison between groups were analyzed by rank-sum test, and the counting data were analyzed by chi square test. *P* < 0.05 means the difference is significant, and *P* < 0.01 means the difference is statistically significant.

## 3. Results

### 3.1. Effect of TAM on the Expression of MLF1IP mRNA in MCF-7 Cells

PCR was used to detect the relative expression level of MLF1IP mRNA in MCF-7 cells treated with TAM to explore the role of MLF1IP in endocrine resistance of Luminal breast cancer.  Figure 1 shows the changes of MLF1IP mRNA expression in MCF-7 cells after TAM treatment. It revealed that the expression level of MLF1IP mRNA in MCF-7 cells was 42% higher than that in the control group treated with PBS after 2 weeks of treatment with 16 *μ*M TAM, and the difference was statistically significant. The results showed that the expression of MLF1IP mRNA in MCF-7 cells was upregulated by short-term TAM treatment, making MLF1IP mRNA highly expressed. The results suggested that MLF1IP mRNA may play a role in the secondary resistance of Luminal breast cancer cells.

### 3.2. Effect of Downregulated MLF1IP Expression on Drug Sensitivity of MCF-7 Cells

MCF7-shRNA and MCF7-NC cells were treated with different concentrations of TAM. The inhibitory rates of MCF7-shRNA and MCF7-NC cells were detected by CCK-8. The effect of MLF1IP on the drug sensitivity of MCF-7 cells was evaluated.  Figure 2 shows the drug sensitivity test results of MCF7-shRNA and MCF7-NC cells. It indicated that the inhibitory rate of MCF7-shRNA and MCF7-NC cells increased with TAM concentration. At different concentration levels, the inhibitory rate of MCF7-shRNA cells was significantly higher than that of MCF7-NC cells. With TAM treatment, the difference in the inhibitory rate between MCF7-shRNA and MCF7-NC cells was of statistical significance (*P* < 0.05). Therefore, downregulating the MLF1IP level of MCF-7 cells could notably increase the sensitivity of MCF-7 cells to TAM.

### 3.3. Role of Cell Proliferation in MLF1IP-Mediated TAM Resistance

It is aimed at excluding the influence of MLF1IP-mediated cell proliferation on the detection of TAM drug sensitivity. 0 *μ*M and 16 *μ*M TAM were selected to analyze MCF7-shRNA and MCF7-NC cell proliferation and the corresponding drug sensitivity (6 groups of repeated experiments under each concentration).  Figure 3 shows the drug sensitivity test results of MCF7-shRNA and MCF7-NC cells. It suggested that the proliferation ability of MCF7-shRNA cells was weaker than that of MCF7-NC cells without TAM (*P* = 0.012). However, under the condition of TAM stimulation, the difference of activity levels between MCF7-shRNA and MCF7-NC cells increased dramatically (*P* < 0.001), and the difference was greater than that of the sum of downregulating MLF1IP alone and TAM treatment alone. These results suggested that MLF1IP-mediated cell proliferation may play a role in the secondary nonspecific resistance of MCF-7 cells, but other factors may be involved in the TAM resistance of MCF-7 cells mediated by MLF1IP.

RETRACTED

### 3.4. Role of Apoptosis in MLF1IP-Mediated TAM Sensitivity

The results above showed that downregulating MLF1IP expression could sharply increase the advanced apoptosis of MCF-7 cells and dead cell population in the usual conditions, while the change of early apoptosis was not apparent. The apoptosis levels of the two groups with ATM treatment were further detected to evaluate the role of apoptosis in the TAM sensitivity of MLF1IP-mediated MCF-7 cells.  Figure 4 shows that the results of this flow cytometry. It was told that after TAM treatment, the late and early apoptosis in both groups significantly increased compared with that under standard culture conditions, and the late apoptosis in MCF7-shRNA cells was markedly higher than that in MCF7-NC cells (*P* < 0.001). Meanwhile, the early apoptosis of MCF7-shRNA cells was significantly higher than that of MCF7-NC cells (*P* = 0.002). Western blot was used in detecting a variety of apoptosis-related proteins to study the relationship between apoptosis and MLF1IP further. The expression of apoptosis-related proteins in MCF7-shRNA and MCF-NC cells with or without TAM was verified at different levels (6 repeated experiments in each group).  Figure 5 shows the detection results of the apoptosis of MCF7-shRNA and MCF-NC cells with or without TAM treatment. It indicated that the expression levels of BAX, Bcl-2, and apoptosis effector proteins (Caspase3, Caspase7, and Caspase9) of MCF7-shRNA and MCF-NC cells had no significant difference. However, after TAM treatment, the expression levels of BAX, Caspase3, Caspase7, and Caspase9 of MCF7-shRNA cells were higher than those in MCF7-NC cells (*P* < 0.05).

In conclusion, under normal conditions, the expression of MLF1IP did not affect the apoptosis level of MCF-7 cells. However, under the stimulation of TAM, the downregulation of MLF1IP could significantly increase the apoptosis level of MCF-7 cells. The results suggested that the apoptosis resistance related to MLF1IP played an essential role in the secondary resistance of Luminal breast cancer cells mediated by MLF1IP.

RETRACTED

### 3.5. Effect of Downregulating MLF1IP on PI3K/AKT Signaling Pathway

The PI3K/AKT pathway was associated with secondary resistance to TAM, the primary therapeutic drug of Luminal breast cancer. The phosphorylation of AKT protein could be induced and promoted by modulating and inactivating PTEN, the tumor suppressor gene in the PI3K/AKT upstream pathway. The phosphorylation of AKT protein could activate the PI3K/AKT pathway and then induce the secondary resistance of TAM. Western blot was used to detect the protein expression related to the PI3K/AKT pathway (6 experiments in each group).  Table 1 and Figure 6 show the detection results. It indicated that the expression of PTEN protein in MCF7-shRNA cells was significantly higher than that in MCF-NC cells (*P* < 0.05), while the phosphorylation level of AKT protein (p-Akt) was lower than that of MCF-NC cells (*P* < 0.05). The results suggested that MLF1IP expression could promote the phosphorylation of AKT and thus activate the PI3K/AKT pathway.

## 4. Discussion

The incidence rate of breast cancer is the highest in the world, and this malignant tumor has become the main reason that affects the quality of life and health of women. Considering the complexity and high heterogeneity of breast cancer, the classification and subtype of breast cancer are determined [10, 11]. In China, breast cancer is divided into Luminal type, ERBB2+ type, and Base-like type. Luminal type is the most common type, accounting for 60%-70% of all breast cancer types [12, 13]. TAM is the main treatment drug for Luminal breast cancer, but during the treatment, many patients will develop resistance to TAM, including primary resistance and secondary resistance [14]. MLF1IP plays an integral part in the pathogenesis of breast cancer and may also be associated with the resistance. In breast cancer cells, the expression of MLF1IP in MCF-7 cells is the highest [15]. Therefore, MCF-7 cells were used to study the molecular mechanism of secondary resistance of Luminal breast cancer based on MLF1IP and TAM.

The results showed that TAM could induce the expression of MLF1IP in MCF-7 cells. Downregulation of MLF1IP could significantly increase the sensitivity of MCF-7 cells to TAM, the endocrine treatment drug. In TAM-treated cells, downregulation of MLF1IP could inhibit the proliferation of MCF-7 cells and promote its apoptosis. The difference between the two groups was more significant than that of MCF-7 cells under normal conditions, which was consistent with the results of Bissoli and Muscari [16]. Western blot results showed that the expression of BAX, Caspase3, Caspase7, and Caspase9 proteins was significantly increased by downregulating MLF1IP in TAM-treated cells, but the expression of Bcl-2 protein was decreased, which matched the study results. Western blot results of PI3K/AKT signaling pathway showed that MLF1IP promoted AKT phosphorylation by inhibiting PTEN expression, thus activating the PI3K/AKT signaling pathway and causing secondary resistance in Luminal breast cancer.

RETRACTED

## 5. Conclusion

The relationship between MLF1IP and secondary resistance of Luminal breast cancer and its molecular mechanism was discussed. The result has shown that MLF1IP plays a vital part in the secondary resistance of breast cancer patients to TAM. MLF1IP promotes AKT phosphorylation by inhibiting PTEN expression, thus activating the PI3K/AKT signaling pathway and causing secondary resistance in Luminal breast cancer. Moreover, MLF1IP can be used as a factor to predict the resistance of Luminal breast cancer to endocrine therapy. The result provided a new indicator for the secondary resistance of Luminal breast cancer patients in the endocrine therapy and a new idea for the treatment of breast cancer.

## Figures and Tables

**Figure 1:** Expression of MLF1IP mRNA in MCF-7 cells after TAM treatment.

**Figure 2:** The drug sensitivity of MCF7-shRNA and MCF7-NC cells (∗compared with MCF7-NC cells, *P* < 0.05).

**Figure 3:** Drug sensitivity test of MCF7-shRNA and MCF7-NC cells (∗∗compared with MCF7-NC cells, *P* < 0.01).

**Figure 4:** Flow cytometry results.

**Figure 5:** Apoptosis level of MCF7-shRNA and MCF-NC cells treated with or without TAM (∗compared with MCF7-NC+TAM cells, *P* < 0.05).

**Figure 6:** Western blot electrophoresis of P13K/AKT signaling pathway-related proteins in MCF7-shRNA and MCF-NC cells.

**Table 1:** Western blot results.

Cell types	PTEN	p-Akt
MCF7-NC	0.34615	2.20512
MCF7-shRNA	0.76923∗	1.03846∗

Note: ∗compared with MCF7-NC, *P* < 0.05.

## Data Availability

Some or all data, models, or codes generated or used during the study are available from the corresponding author by request.
